# Analysis of Legal Issues of Personal Information Protection in the Field of Big Data

This article has been retracted.

**DOI:** 10.1155/2022/1678360

**Published:** 2022-08-29

**Authors:** Chuyun Wang, Feifei Guo, Mengxuan Ji

**Affiliations:** ^1^Central University of Finance and Economics, Beijing 100081, China; ^2^School of Medicine and Humanities, Capital Medical University, Beijing 100069, China; ^3^School of Public Administration, Xi'an University of Finance and Economics, Xi'an, Shaanxi 710100, China

## Abstract

In the era of big data, while every citizen enjoys the convenience of the Internet, all kinds of information closely related to their personal and property are in a state of “streaking” for a long time. Personal information is frequently leaked, illegally misappropriated, and used. There are necessary requirements of network security. The risks and challenges faced by personal information in the context of big data increase. In the context of the rapid development of big data, the information is circulated in virtual cyberspace in the form of electronic data, and data sharing has become an important flow form of information circulation. It is an important link to realize the optimal allocation of network resources and realize the value of data. The great progress of the digital economy and artificial intelligence technology has greatly increased the demand for data, the speed of circulation has been further accelerated, and the potential value of data has been fully reflected. At present, the scope of personal information protected by Chinese laws is relatively narrow and is basically limited to the scope of privacy rights, which makes a large amount of information owned by individuals that do not belong to the category of personal privacy rights lack legal protection. Personal information is different from the characteristics of privacy rights. It is decided that the protection of personal information should be different from the protection of traditional personal privacy. To sum up, in view of this, this article attempts to analyze the new challenges faced by personal information protection in the era of big data from the perspective of law, combined with the background of the era of big data, from the legislative model, system design, supervision mechanism, industry self-discipline, and other aspects. Exploration of the legislative framework for the protection of personal information in the era of big data in our country is done in order to find a realistic path that balances the development of big data technology and the protection of personal information.

## 1. Introduction

In recent years, with the popularization of the Internet, people's life style has entered the era of mobile Internet and all things interconnected. In just a few short years, the amount of information that exploded has accumulated enough to spark a revolution. A huge amount of data is generated in various fields at the same time. The amount of data has exceeded the limit of traditional data analysis and processing tools. This has prompted the emergence of new technologies to process and analyze excess data, which is the origin of big data. The advent of the era of big data has completely changed people's concept of data. Facebook, the largest social company in the world, has billions of users, more than tens of millions of pictures are uploaded by users every day, and the number of followers and comments exceeds 3 billion people every day. YouTube, the world's largest online video site, has more than 1.5 billion monthly viewers and hundreds of thousands of videos are uploaded every second. Google generates more than 24 petabytes of data every day, which is far more than any traditional data processing organization on the planet. From scientific research to everyday life, there is an explosion in the amount of data in all the different fields that humans dabble in. If such a huge amount of data is used in traditional ways, it will cause great waste and cannot generate enough value. Through big data technology, by analyzing massive amounts of data, it is possible to obtain sufficiently accurate predictions. Such accurate predictions about the unknown can make revolutionary changes in all walks of life [1–5].

However, with the advent of the era of big data, many problems that did not exist before also arise, especially the protection of personal information. In the era of big data, the nature of the threat posed by the breach of personal information has changed. The role of personal information data is no longer limited to its initial purpose but can generate new value in the process of its secondary or even multiple use. This challenges the individual-centered thinking under current personal information protection laws. Under current law, data collectors must inform individuals about what data they collect and for what purpose, and they must also obtain their consent before collection begins. In the era of big data, a lot of data is only used to complete a certain job when it is collected, but in the end it has many unexpected uses through multiple utilization. The data collectors themselves cannot even fully anticipate the value and effects of the collected data. And what if every use of the data is temporarily notified for use? In the era of big data, traditional notification and permission are outdated. Either it is too narrow, and the mining of the potential value of big data will be idle; or it is too general, making the protection of personal information an empty talk. In August 2015, the State Council issued the “Outline of Action for Promoting the Development of Big Data,” which formally proposed to “implement the National Big Data Strategy.” The outline proposes three major tasks. The first is to speed up the opening and sharing of government data, promote the integration of resources, and enhance the government's governance capabilities. The second is to promote the innovative development of the industry, cultivate emerging industries, and accelerate the transformation of the economic structure. The third is to strengthen security, improve management, and ensure healthy development. In addition to the three major tasks, the outline has raised the development of big data to the height of the strategy of strengthening the country, established the core concept and management mechanism of China's big data development, and planned ten key projects and a series of national and regional big data platform construction. Task: Promoting the development and application of big data has become the core strategy of the country. The issue of personal information protection has received unprecedented attention. In the era of big data, information has become a resource, and its universality, sharing, value-added, and processability make it practical and practical, especially personal information, which includes not only personal privacy, but also all the information left by personal activities. Through the mining and utilization of this information, it can provide great help to the government and enterprises in decision-making and management. However, due to the lack of an effective personal information protection mechanism, there are serious information security problems in our country. Economic losses and personal safety violations caused by personal information leakage are not uncommon in China. In this context, calls for strengthening the protection of personal information are growing. At this year's National Two Sessions, many representatives suggested that the implementation of the Personal Information Protection Law should be accelerated to strengthen our country's personal information protection. The amount of data in the billions and megabytes makes the job nearly impossible if the user agrees. And if the user agrees to all possible uses of the data in advance, then there is no point in talking about the protection of personal information.

## 2. Related Work

Big data technology has now been applied to most industries and is an indispensable and important production factor. What big data brings to all walks of life is not only a new data technology, but also a complete revolution of the entire system. Through the mining and application of massive data, a new wave of productivity growth and consumer surplus is coming. After 2007, with the comprehensive development of the Internet and the rise of social networks, the era of the Internet for the whole people has gradually arrived, and big data has gradually become a popular word in the Internet technology industry. In 2009, the US government launched the government data website and began to open the door to data. In June 2011, McKinsey released a report on “big data” “Big Data: The Next Frontier of Innovation, Competition and Productivity,” which pointed out that “the era of big data has arrived.” This report has received high attention from all walks of life. Since 2017, big data has entered all aspects of people's lives. Under the combined force of multiple factors, the big data industry has ushered in explosive growth. Up to now, more than 13 provinces across the country have established 21 big data management institutions. Among colleges and universities across the country, 293 schools have applied for undergraduate majors in data science and big data technology. At the same time, a series of heavyweight global conferences such as the World Economic Forum in Davos in 2018 took “big data” as an important topic and conducted a comprehensive discussion and analysis of it. The wave of big data development is sweeping the world. According to statistics, the total amount of data in the world in 2017 was 21.6ZB (1ZB = 1,073,741,824TB), and this amazing amount of data is still growing rapidly at a rate of 40% per year, as shown in Figure 1 [6–13].

We can see that the real rise of big data started from the Internet era. The emergence of a variety of emerging information technologies provides solid technical conditions for big data. The best example is the variety of portable connected devices (smartphones, smart glasses, smart bracelets, etc.). The emergence of various technologies and products provides a guarantee for the recording, uploading, and application of massive data. In the past ten years, a large number of high-tech companies represented by Goggle have successively entered the field of big data and achieved great success in it, turning big data technology into practical business results. In this process, the public also quickly realized the important role of big data technology, driving more industries to invest in the research and development of big data. Big data can be said to be an inevitable product of the development of information technology. With the development and maturity of the Internet and the continuous expansion of application fields, the total amount of data generated continues to increase. In the process of trying to use these data, big data came into being.

Compared with other disciplines, “big data” is a very young thing. It has only been thirty or forty years since it was proposed. But for the definition of big data, there is currently a lack of a recognized, unified, and absolute standard. From the perspective of the amount of data, the amount of big data must be at least too large to be processed by conventional tools and conventional methods, requiring the use of specific tools and models. The level of data volume varies for different industries. As far as big data itself is concerned, it is a huge, almost infinite collection of data, the sum of data in a field or fields. But when we discuss big data, we find that it refers more to big data technology or to discussing its concepts at a technical level. Of course, it is undeniable that when we use the term “big data,” we often have both concepts. Therefore, there are many opinions in the academic circle about the characteristics of big data. Among them, the most widely supported are “3 V” and “4 V.” Among them, “3 V” is the three characteristic elements of big data development proposed by Doug Laney, an analyst at Meta Group in 2001, namely, Volume, data capacity is getting bigger and bigger; Velocity, data processing speed is fast, and growth is fast; Variety, more and more types of data. Then, with the development of big data, Value was added on the basis of “3 V,” and the value density was low, forming the most widely accepted “4 V,” that is, large data capacity, various types of data, and data processing. With the development of big data, the complexity of data is getting higher and higher, and some people keep making the assertion of new characteristics of big data, which has developed to 5 V (increasing Veracity is low in accuracy), 6 V (increasing Vitality is high in dynamics), and even 7 V and 8 V. But today, the 4 V argument is still the most accepted by the academic community, as shown in Figure 2 [14].

The data capacity is large. The biggest feature of big data is undoubtedly the huge amount of data, which needs to be discussed at least in terabytes or petabytes. This level of data volume has completely surpassed the scope of traditional statistics. It cannot be analyzed using traditional analysis tools and models. In the past, when faced with huge statistical data, because we could not use all of them, we could only select a part of random samples, analyze the samples, and draw conclusions. In the era of big data, we are not just analyzing a part of the data of a random sample, but all the data related to something. Big data has various data types. Traditional data statistics can only analyze structured data. According to IDC statistics, 80% of the data in enterprises is unstructured data. Big data can make full use of structured data, semistructured data, and unstructured data for analysis and statistics. Data processing is fast. In traditional statistics, it takes a long time to collect data, input data, and analyze data, and the results often have a certain lag. And for big data because its data is always online, and a large amount of data is generated every day, first of all, it reflects the rapidity of big data data generation. Through the calculation of powerful servers, it can ensure the timely processing of massive data and ensure the value of data and conclusions. Data has high value and low value density. Because of its huge data capacity and various types of information, big data has a very high value. However, the high value of big data is based on its huge data capacity, and its value density is very low. The data with direct value is often only a small part, and most of the data has no value or requires a very complex model to produce a certain mechanism. Therefore, only cloud computing, which integrates dozens, hundreds, or even thousands of computer analysis capabilities, can complete the analysis of massive data. In addition to the traditional “4 V,” big data also has an important feature that is “Online,” which is always online. Data is generated and recorded instantly. All data is online in real time, rather than being generated after statistics.  Figure 3 shows the big data warehouse model.

## 3. Special System Design for Personal Information Protection in Big Data Environment

Human society entered the era of big data, and big data technology itself is still developing rapidly. The lag of laws is particularly prominent in this field. The current situation and trends of big data development have also had a great impact on personal information legislation. The characteristics of big data, such as large capacity, fast update and iteration, and cross-domain, make the American style decentralized legislation more and more powerless. In the early days of information technology development, the number of websites and applications was relatively small and relatively independent. A single data set was often managed corresponding to a specific field, and cross-field data rarely appeared. In the era of big data, taking China as an example, the subsidiaries and investment companies of Internet giants such as Alibaba, Tencent, and ByteDance basically cover all aspects of life. Many traditional manufacturing and service industry giants such as Suning and Gree have also developed the Internet. In industries such as finance and smart home, the complexity of personal information data is not comparable. At the same time, new sources of big data services, such as group purchases, shared bicycles, online taxis, and time-sharing, have emerged one after another in recent years. The rapid development of big data and the accompanying complex and changeable forms of personal information cannot be enumerated by separate legislation. The model of decentralized legislation in the United States is obviously unworkable under big data. The leakage of personal information under big data has also undergone tremendous changes, posing new challenges to legislation. For example, the frequency of personal information leakage incidents continues to accelerate, and even with complete legal support, it is difficult to achieve real-time monitoring, discovery, and processing. It is imperative to establish a special personal information regulatory agency; the number of personal information leakage subjects is also increasing. In the traditional data society, large-scale personal information is only stored in the government, and enterprises store a limited amount of user information in separate segments. For example, in the fight against the new crown epidemic in early 2020, Alipay and the government launched a health code service to cooperate with citizens' network footprints, which can well achieve the effect of monitoring and predicting the epidemic; the way of personal information leakage has also become more diverse. Traditional data leakage mostly occurs in hackers, Trojan links, etc. In the big data environment, the abuse of cookies (small text files) leads to more personal information leakage. This technology can record user behavior on the page, directly steal user account password and other information, and track it. The above points make personal information infringement more concealed in the big data environment, and the status of the perpetrator and the victim becomes more and more unequal, which requires special attention in legislation [15–18]. Personal information protection legislation in the era of big data cannot be limited to the traditional protection of personal information from leakage and the obligation of the government and information collectors to protect personal information. Focusing on the current international situation and technological trends, personal information protection legislation should have new and unique system designs in the development and utilization of personal information, national security, and remedies.

### 3.1. The Introduction of the Long-Arm Jurisdiction System

For a long time, domestic personal information legislation has followed the principle of territorialism. Only information collected in China or data equipment set up in China is under the jurisdiction of China. However, when the society enters the era of big data, especially after the emergence of cloud computing, a large part of personal information, business data, and even government data are processed in cloud computing, and the phenomenon of cross-border data flow is increasing. However, differences in politics, economy, and law will inevitably lead to games between countries on personal information, and countries have also strengthened the management of cross-border data. The 2016 EU General Data Protection Regulation innovatively stipulates that all matters involving the personal information of EU citizens can be governed by GDPR, known as long-arm jurisdiction. This means that all suppliers providing services to EU citizens, whether their establishments, equipment, and personnel are located in the EU or not, are subject to the GDPR. This clause becomes a worldwide clause when personal information involves the EU, which greatly increases the right to speak in personal information affairs in the EU. China can draw lessons from the long-arm jurisdiction of GDPR when legislating personal information. Although this does not mean that China should take the initiative to provoke personal information disputes, at least China has corresponding legal endorsements when cross-border information disputes arise, which can better guarantee the development of China's big data economy.

### 3.2. Outbound Management of Personal Information

The cross-border flow of personal information in the era of big data has become a trend, but the exit of personal information will cause many security risks: First, after personal information is stored overseas, there will be security breaches and hacker attacks in the information of overseas information storers. The personal information of Chinese citizens is easily transferred, sold, and used illegally. In recent years, there have been frequent cases of personal credit cards being stolen overseas; that is, the names, phone numbers, information card information, etc. that were saved when citizens stayed overseas were leaked; second, personal information was subject to local laws and regulations after leaving the country. However, many countries still do not have mature personal information laws and regulations, and the jurisdiction of personal information in many developed countries is limited to their own residents. Once personal information is violated, Chinese citizens may not be able to claim their legitimate rights and interests; third, once the incident occurs in the event of personal information infringement, it is very difficult for Chinese citizens to obtain information within the country, and they may not know that their rights and interests have been infringed. Even if the information subject knows the occurrence of the infringement, it is very difficult to obtain evidence. It is not uncommon for it to be installed overseas and the network transmission path passes through overseas. Most personal information subjects are unaware of this, and network operators have not fulfilled their due reminder obligations. In the big data environment, the cross-border dissemination of personal information data is unavoidable, and it is obviously not in line with the trend of the times to restrict and monitor the online cross-border behavior of personal information subjects. However, from the perspective of national security and personal information protection, in order to prevent a large number of Chinese citizens' information from being obtained overseas, it is still necessary to supervise the cross-border data flow of network operators [19]. For example, a predeclaration system for network operators can be established to report to the regulatory authorities in advance the scope, method, and purpose of outbound personal information. After review and approval, you can leave the country, establish personal information exit file management, and keep all exit information for the record.

### 3.3. Protection of Children's Personal Information

In the era of big data, a large number of children with immature minds can easily access smart network devices. As a result, it is not uncommon for children's personal information to be illegally collected and used by Internet operators or other harmful subjects, causing great harm to children and their families. Respecting and protecting children's rights is a widely recognized basic knowledge, and the protection of children's personal information has also been gradually introduced into the personal information protection laws of various countries. The Children's Online Privacy Protection Act of the United States and the EU GDPR both stipulate the age division of children's personal information, the verification of children's age, and the guardian's permission system. However, there is no separate legislation for children's personal information network security in China at present. In the unified personal information protection legislation, the following rules can be used to protect children's personal information: First, set up special children's personal information protection rules and user agreements, designate a person to be responsible for the protection of children's personal information, and control the authority to obtain such information from internal controls. The information controller should distinguish between the user agreement and the privacy service agreement between adults and minors and should set up a special person to be responsible for the protection of children's personal information. In addition, due to the particularity of children's personal information, the company should also establish a complete acquisition and access authority system and strictly control the number of people who acquire and access such children's information. Second, inform the guardian of the child in a conspicuous and clear way, the consent of the guardian of the child should be obtained, and the option of refusal should be provided. Although there is currently no 100% effective method to identify “real” adult or minor users, at least for those users who directly use minors' ID information, information controllers need to arrange and deploy corresponding technical solutions. For example, an account registered with a minor's certificate needs to be bound to the e-mail or mobile phone of its guardian, and verification information is sent to the guardian's mailing address during registration to remind him to make a second confirmation. At the same time, the information controller shall provide the guardian with the option of “rejection” when performing the technical settings agreed by the guardian. Third, provide ways to make complaints and reports and how to correct and delete children's personal information. The information controller shall set up a complaint and report channel to receive complaints and reports from users and promptly respond to users' requests for correction and deletion of children's personal information that is incorrect or without the consent of the guardian.

### 3.4. The Introduction of the Right to Be Forgotten System

The right to be forgotten, i.e., the right of the data subject to ask the data controller to delete personal data about him: the controller has the responsibility to delete the personal data in a timely manner in specific circumstances. The concept of the right to be forgotten is well known in the Gonzalez v. Google case before the Court of Justice of the European Union. Doctor Gonzalez asked Google to delete negative news about him from relevant search pages. Right to forget: The EU formally enshrined the right to be forgotten in its GDPR in 2016. Many scholars refer to the right to be forgotten as the right to erasure of personal information, and this study argues that the right to be forgotten is different from the right to erasure. The usage scenario of the right of deletion is that when the information is illegally collected and utilized, the subject of the right can delete the information involved by exercising the right of deletion. The focus of the right to be forgotten is to exclude the relationship between the information and the subject of the information. The relevant information does not have to be deleted. The effect of exercising the right to be forgotten can also be achieved by means of information correction, lowering the weight of search results, and information anonymity. It can also be deleted when invalid. Deletion as a way of realizing the right to be forgotten is ultimate and humble. As Tencent's privacy policy states, “Even if you delete shared information, the information may still be independently cached, copied or stored by other users or unaffiliated third parties that are not under our control, or shared in public by other users or such third parties. Domain Preservation.” Such information can only be adjusted by the right to be forgotten. The right to be forgotten is typical new rights and interests that have emerged due to technological development, and there are many debates on the right to be forgotten. For example, for subjects who exercise the right to be forgotten, if everyone can exercise the right to be forgotten to delete their past records in the large database, it will inevitably cause moral hazard; whether the right to be forgotten is inconsistent with the characteristics of open circulation of big data information, and where is the boundary for exercising the right to be forgotten? [20] For these issues, this study believes that the right to be forgotten can be exercised if the following conditions are met: first, the prepurpose of the information collector using personal information has been achieved; second, the authorization of the personal information right holder is time-limited and the limitation period expires; third, the personal information is collected illegally or falsely by the information collector.

### 3.5. Right to Portability of Personal Information

The right to portability of personal information means that the subject of personal information has the right to obtain the information provided by the information controller (must be generalized and machine-readable) after providing the information to the information controller and has the right to transfer his data to other controllers. It is a legitimate right of users to authorize their personal data information on a certain platform to be used by other platforms. In daily life, allowing software to read the address book and use WeChat to log in to other software is manifestations of the right to information portability. The right to information portability may seem simple, but there are many disputes between academia and big data companies. The reason is that the use of personal information is likely to also involve other third-party personal information, such as address book information, e-mail exchange information, transfer record information, etc. When the information subject exercises the right to information portability, it may often infringe the basic rights of other third-party individuals. For example, in 2010, when Google launched its social networking service Google buzz, it improperly used the relationship chain data of its gmail users. When a gmail user accepted an invitation to use Google buzz, it was not clear who was in the address book of his gmail. Users who are pulled in will not know that their contact information has been included and made public by the buzz community. Google has also been punished by the US Federal Trade Commission. The right to information portability is a right arising from the flow of user information, but the flow of information is also the competitive advantage of big data. A series of problems arising from the flow of information should be stipulated in the personal information protection legislation, and the information controller restrictions and penalties are imposed on the use of information flow and unreasonable market competition. Information under big data has become a kind of commercial capital and an important economic investment. The acquisition and use of data can not only become a source of competitive advantage for enterprises, but also create more economic benefits for enterprises, which is an important factor for operators. With competitive advantages and commercial resources, the protection of the right to information portability can be regulated with reference to the relevant provisions in the Anti-Unfair Competition Law. [21].

### 3.6. Handling of Large-Scale Information Leakage

In the traditional data era, only the government can store a wide range of citizens' personal information. Because of the narrow information collection field and the small target user range, the personal information leakage of enterprises is characterized by small scale, specific information, and small dissemination scope. However, in the era of big data, leading Internet companies have also mastered a large amount of personal information. For example, the number of monthly active users of WeChat in 2019 has reached 1.151 billion, and there are nearly 100 applications with more than 100 million monthly active users in China. If the information databases of these companies are leaked, the scale and severity are unimaginable. For example, in 2018, the Huazhu Group database was stolen, and nearly 500 million pieces of user information were packaged and sold on the dark web by hackers, including user names, credit card information, check-in records, etc. The current large-scale information leakage incidents are characterized by many data subjects, wide data content, strong dissemination, and serious follow-up impacts. But the relief of China's current legislation for large-scale data breaches is insufficient. Personal information infringers (hackers, hacker organizations, etc.) are often left behind because of the difficulty of tracking and the difficulty of jurisdiction in other countries' territories; for the information users of the leaked data information, they can only order them to repair loopholes to strengthen supervision or administrative fines and other penalties; and for victims of massive personal information leakage, the remedies are very limited.

## 4. Market Supervision and Industry Self-Discipline of Personal Information in Big Data Environment

### 4.1. Overseas Personal Information Market Supervision and Industry Self-Discipline

Personal information protection legislation in the United States is scattered and basically falls within the scope of personal privacy protection. The United States, which corresponds to the legislation, has a strong industry self-discipline protection mechanism. In July 1995, the US government's Privacy Protection Working Group first issued “Personal Privacy and the National Information Infrastructure: Principles for the Use and Provision of Personal Information,” which first stipulated a set of common benchmarks for regulating personal information self-discipline. In July 1999, the US Federal Trade Commission believed that the best choice to protect individuals' discretion is to test highly effective industry self-discipline, which pointed out the direction for further encouraging and guiding the industry to implement self-discipline. For example, the American Internet Business Alliance has issued the “Internet Privacy Protection Self-discipline Guidelines” and set up a special online privacy certification system. Only certified websites and software will be identified to distinguish them from other websites and software; network operators only need to comply with industry self-discipline guidelines; there are certain disclaimers after the time of personal information leakage, etc. The EU “Personal Information Protection Directive” requires EU member states to set up a separate personal information protection center, with a special personal information affairs processing specialist, with full professional power to handle supervision and law enforcement affairs related to personal information. This can better protect citizens' personal information. In the field of private rights, the GDPR stipulates that information controllers and processors should appoint a special information protection officer, whose main functions are as follows: provide personal information-related advice to information controllers or processors; information-related policy compliance review and employee training; act as a liaison for information control and processors, and connect with the personal information protection center. Japan's “Personal Information Protection Law” and its 2015 amendments set up a special personal information protection committee, which is also responsible for personal information protection and personal information supervision. However, unlike the European Union, the committee does not belong to the referee management agency, but only for consultation. Organizations, which are not government agencies and have a high degree of autonomy, reduce the interference of government powers on personal information and protect citizens' freedom of personal information in the field of public powers. Under the guidance of the Personal Information Protection Committee, industry self-discipline guidelines will be established in various industries to protect personal information from being abused and stolen in the field of private rights. The Japan Information Processing and Development Association has issued the “Guidelines for the Protection of Personal Information in the Private Sector” and the corresponding requirements “Requirements for the Management System of Personal Information Protection (JISQ15001).” Accordingly, JIPDEC starts the corresponding evaluation certification, and the companies that pass the evaluation will receive the corresponding grade certificate.

### 4.2. The Choice of China's Personal Information Market Supervision System

In the era of big data, the development of big data industry technology and the protection of personal information are contradictory to a certain extent, and the ever-changing technological iterations make it more difficult to find a balance between the two. On the other hand, the follow-up of the legislative systems of foreign countries, such as the implementation of the EU GDPR long-arm jurisdiction principle, has made many domestic network service providers turn to meet EU standards to carry out the collection and use of personal information. China urgently needs to establish a complete market supervision mechanism to protect the personal information security of domestic citizens, maintain national security, and promote the development of the big data industry. A market environment that is too strict or too loose has drawbacks. This study believes that China should establish a model with market supervision as the mainstay supplemented by industry self-discipline. [22].

#### 4.2.1. Establish a Personal Information Market Supervision Department

The actual supervision of China's current big data market, the leakage and abuse of personal information in China is serious at present, and most of the existing personal information clauses appear in normative documents. To deal with personal information security incidents in a timely manner, the remedies for personal information rights holders and the penalties for infringing parties are not in place. In this case, it is necessary to set up a unified market supervision agency to change the market chaos. At the same time, a personal information supervision agency with clear functions and powers is conducive to coordinating personal information protection measures in different industries and fields and effectively and orderly balancing personal information protection and large-scale development of the data industry. As of September 2019, China has established 16 provincial-level big data management institutions and 22 big data management institutions below the provincial level and initially established a big data bureau to manage and formulate data resource collection, governance, sharing, and openness in the setting of administrative institutions, application, security, and other technical standards and management methods, to achieve cross-level, cross-department, cross-system, and cross-business data sharing and exchange. This shows that the government has fully realized the importance of big data, and the establishment of specialized agencies can really urge all departments at all levels to pay more attention to the construction of big data.

#### 4.2.2. Formulate Technical Standards for Personal Information Protection Security

At present, the domestic technical standards for personal information protection are mainly the “Information Security Technology Personal Information Security Specification” issued and revised by the State Administration for Market Regulation and the National Standardization Administration. Behaviors and handling of personal information security incidents provide certain behavioral templates, as well as suggested templates for personal information use agreements. However, no clear technical standards have been given for more detailed technical details such as personal information storage and encryption. In the past two years, mobile apps have not dealt well with problems such as excessive requests for permissions and unauthorized activation. Therefore, it is necessary for our country to formulate and improve truly effective technical standards for personal information protection and security in light of the new situation of constantly developing big data, closely following the market and technology. Our country has always had a tradition of overly strict government supervision. Therefore, when setting up market supervision mechanisms and formulating technical standards, we also need to pay attention to the following points: First, it is necessary to control the collection of citizens' personal information by government agencies and other information collectors. Personal information, especially sensitive personal information, should be carefully collected and have a complete supervision and filing mechanism, and the government should be restricted in the field of public power to better protect the freedom of citizens' personal information; second, Internet big data companies are exposed to personal information. When formulating policies, market regulators should take into account market conditions and listen to the opinions and experiences of market players, so that personal information protection policies can be truly implemented.

### 4.3. The Establishment of Self-Discipline in China's Personal Information Industry

In the era of big data, overly strict market supervision is not conducive to the healthy development of the market. On the basis of unifying personal information legislation and establishing market supervision institutions, the reasonable application of big data personal information should be appropriately relaxed, and on the basis of personal information protection it allows citizens to better enjoy the convenience of life brought by big data and can also promote the continuous development of big data technology and industry. In recent years, a large number of international technology-leading companies such as Alibaba, Tencent, and ByteDance have emerged in China. The government has also carried out in-depth cooperation with Alipay and WeChat. Internet convenience measures and online government affairs halls have achieved good results. Many personal information protection groups or industry exchange forums have also been established within or among Internet companies [23].

#### 4.3.1. Establish the Legal Status of Industry Self-Regulatory Organizations and Their Guidelines

The US “Children's Online Privacy Protection Rules” stipulates that the industry guidelines approved by the Federal Trade Commission can be regarded as laws, and our country can learn from this. Industry self-regulatory organizations approved and established by government regulatory authorities can obtain independent legal person status in accordance with the law, and the articles of association and industry standards formulated by them can also be binding on practitioners. In light of the specific national conditions, it is necessary for our country to clarify the relationship between government regulatory agencies and specialized industry associations. Regulatory agencies can exercise overall control over the market by regulating industry regulations and establishing technical standards for personal information protection, with actual feedback from the market, combining policy formulation with market reality.

#### 4.3.2. Establish an Industry Self-Discipline System

Government regulatory agencies and industry self-regulatory organizations should establish stricter industry self-discipline standards on the basis of laws, regulations, and market supervision with the consent of members. For example, the network information privacy logo is advocated, and web pages and applications that meet the network privacy security certification can use this logo to facilitate user identification and establish a green application alliance to encourage mutual supervision and incentives among industry members, so that practitioners do not respond to laws and regulations. To take personal information protection measures according to regulations, so that excellent personal information protection companies can gain more exposure and public recognition, with anonymous data review, promote all big data to be displayed anonymously in the cloud, and network service providers can only perform operations on a wide range of big data. Analysis of region, age, frequency, etc. cannot accurately analyze specific individuals, etc. Strict industry self-discipline standards can, on the one hand, better protect the security of personal information and prevent personal information security incidents; on the other hand, it will help high-quality companies gain better market recognition and keep the big data industry in a virtuous circle.

#### 4.3.3. Establish a Data Commissioner System

The data commissioner system should be promoted in big data enterprises. A full-time department or employee is responsible for connecting with the personal information regulatory agency and regularly reporting the company's information protection measures, whether there is a risk accident, etc.; the data commissioner should provide the enterprise with professional advice on personal information matters and participate in any process involving the collection, utilization, and storage of personal information. In corporate affairs, conduct compliance reviews on corporate personal information-related activities, conduct regular corporate risk self-examinations, and conduct regular employee training, etc.

#### 4.3.4. Establish a Third-Party Evaluation Mechanism

Personal information protection in China started late, and there is currently no authoritative organization to evaluate and test personal information protection capabilities. In this case, it is urgent to establish a sound third-party evaluation mechanism. First of all, there must be complete personal information protection standards for information subjects and information collectors to check and self-check; secondly, improve the operation system of third-party evaluation agencies and establish a personal information security accident early warning, relief, and stop loss system, and professional policy guidelines are given regularly.

#### 4.3.5. Standardize the Personal Information Use Agreement

The authorization of network service providers to obtain users' personal information comes from the privacy agreement. However, for a long time, the privacy agreement entry is hidden, the privacy agreement is merged into the user agreement, and the agreement requires unreasonable permissions. The problem is very serious, and many users have given permission without knowing it. Unreasonable collection and use of personal information: “The privacy clauses of 47 apps are not up to the standard, and 34 apps have no privacy clauses.” The China Consumers Association conducted an evaluation of 100 mobile apps in 2019 and found that the abuse of mobile app usage rights and the substandard privacy clauses may cause user privacy leakage. In addition, the “Investigation Report on APP Personal Information Leakage” released by the China Consumers Association shows that 85.2% of the respondents have been harassed or violated due to personal information leakage. In response to this phenomenon, in December 2019, the Cyberspace Administration of China, the Ministry of Industry and Information Technology, the Ministry of Public Security, and the State Administration of Supervision jointly issued the “Methods for Identifying the Illegal and Illegal Collection and Use of Personal Information by Apps,” which made many provisions on this. The purpose, method, and scope of the collection and use of personal information, the collection and use of personal information without the user's consent, the violation of the principle of necessity, and the collection of personal information irrelevant to the services provided are all identified. In addition, this study believes that the term “privacy agreement” should also be changed to “personal information use agreement,” because the scope of personal information is far greater than personal privacy, and the legal and reasonable use of personal information and personal privacy are guaranteed in the era of big data. Not being infringed is equally important, and it should be attributed to the management of the personal information use agreement.

## 5. Conclusion

Compared with traditional personal information protection in the era of big data, it is more difficult to determine the infringing subject, the infringing acts are more diverse, and personal information is more likely to be illegally obtained, sold, or even illegally committed. However, our country's personal information protection is obviously insufficient; there are problems such as scattered laws and regulations, poor operability, vague definition of personal information, imperfect informed consent rules, immature rights relief mechanism, insufficient administrative protection, and lack of criminal law protection.

In view of the problems existing in the protection of personal information in the era of big data, special legislation can be formulated and the industry self-discipline mechanism can be improved to balance the relationship between the protection and utilization of personal information. At the national level, first, formulate a personal information protection law. In terms of specific content, introduce scenarios and risk assessment mechanisms, attach importance to the protection of personal information in the process of using it, clarify the definition of personal information, improve the legality rules for information collection, enrich the content of the rights of the information subject, and optimize the rights relief mechanism; secondly, set up a special supervision agency to strengthen the supervision of the use of personal information, and regulate the rational use of personal information by government personnel, with punishment for major related crimes. At the social level, improve the industry self-discipline mechanism, clarify the legal status of industry self-discipline in law, formulate relatively complete industry self-discipline norms, set up industry certification bodies, and gradually realize the comprehensive protection of personal information.

## Figures and Tables

**Figure 1:** Global data generation and forecast (Source: IDC).

**Figure 2:** Big data feature map.

**Figure 3:** Big data warehouse.

## Data Availability

The dataset can be accessed upon request.
